# Comparison of Oral versus Intravenous Proton Pump Inhibitors in Preventing Re-bleeding from Peptic Ulcer after Successful Endoscopic Therapy

This article has been retracted.

**DOI:** 10.7759/cureus.6741

**Published:** 2020-01-22

**Authors:** Rashid Karim, Rizwan Hameed, Kashif Ali, Amber Tahir

**Affiliations:** 1 Gastroenterology, Dera Ghazi Khan Medical College and Hospital, Dera Ghazi Khan, PAK; 2 Internal Medicine, Dera Ghazi Khan Medical College and Hospital, Dera Ghazi Khan, PAK; 3 Internal Medicine, Dow University of Health Sciences, Karachi, PAK

**Keywords:** route of administration, proton pump inhibitora, pantoprazole, rebleeding, recurrent gastrointestinal bleeding, peptic ulcer disease, endoscopy

## Abstract

Introduction

Perforation, obstruction, and bleeding remain the most frequently encountered complications of peptic ulcer disease (PUD). Bleeding may be in the form of hematemesis or melena. The treatment of choice in patients with a bleeding peptic ulcer is endoscopic ligation to maintain the hemostatic balance followed by the administration of proton pump inhibitors (PPIs). This study focuses on the evaluation and comparison of intravenous (IV) and oral PPIs in terms of prevention of re-bleeding after successful endoscopy for peptic ulcers.

Methods

A prospective, comparative study was conducted in a tertiary care hospital in Pakistan from January 1, 2018 to June 30, 2019. The trial included known cases of PUD admitted with active upper gastrointestinal bleeding (UGIB). They were randomly divided into two groups: one received oral pantoprazole and the other was administered IV pantoprazole. The outcomes for both groups were compared. Data was entered and analyzed using Statistical Package for the Social Sciences (SPSS) software version 23.0 (IBM, Armonk, NY)

Results

There were 96 (48%) patients in the IV pantoprazole group and 104 (52%) in the oral group. From 24 hours after the medication onwards, the IV pantoprazole group showed a significant improvement in hemoglobin (Hb) levels (p: 0.01); the group also showed improvement in supine systolic BP at 48 hours (p: 0.04) and in diastolic BP at both 12 and 48 hours as compared to the oral pantoprazole group (p: 0.05). The mean duration of hospital stay, need for blood transfusion and repeat endoscopy, re-bleeding, and mortality rates were similar for both groups (p: >0.05).

Conclusion

We could not find any statistically significant difference between oral and IV routes of pantoprazole administration in the prevention of rebleeding when used after successful therapeutic endoscopy in patients with bleeding PUDs.

## Introduction

Peptic ulcer disease (PUD) is a multifactorial condition; it may be caused by various factors such as gastric acid hypersecretion, dietary habits, psychological stress, Helicobacter pylori (H. pylori) infection, and chronic use of nonsteroidal anti-inflammatory drugs (NSAIDs). Perforation, obstruction, and bleeding remain the most frequently encountered complications of PUD [1]. Bleeding may be in the form of hematemesis or melena. Over the years, the incidence of upper gastrointestinal bleed (UGIB) secondary to PUD has declined due to earlier diagnosis made possible by the advancements in endoscopy, therapy adherence, and successful treatment of H. pylori [2]. However, UGIB still remains the most common complication of PUD and often causes morbidity and mortality in patients [1,2]. The treatment of choice in patients with a bleeding peptic ulcer is endoscopic therapy to maintain hemostatic balance. Endoscopy reduces the requirement of surgery, risk of re-bleeding, and rate of mortality in such patients. [3]. Despite being a very successful and useful mode of treatment in bleeding peptic ulcers, chances of re-bleeding in patients after endoscopic therapy are still as high as 14-36% [4].

The role of gastric acid in the stomach and duodenum is to inhibit the formation of clots. Excess acid secretion results in lysis of clots and thereby increases the chances of bleeding [5]. Hence, reducing gastric acid secretion helps in reducing the chances of bleeding in patients with PUD [6,7]. The most commonly used drugs for reducing gastric acid secretion are proton pump inhibitors (PPIs). It has been suggested that intravenous (IV) and oral PPIs are comparable in efficacy in PUD patients [8]. Higher doses of oral PPIs act faster and are more effective in acid suppression. However, higher doses of IV PPIs are more effective than high doses of oral PPIs [9]. Despite extensive research and advancements in therapy, the optimal dosage and route of PPIs administration after endoscopic therapy to prevent re-bleeding of peptic ulcers is still a matter of controversy. Most previous studies did not find any significant difference between the efficacy of IV and oral PPIs after endoscopic therapy to prevent re-bleeding of peptic ulcers. This study focuses on the evaluation and comparison of IV and oral PPIs in terms of prevention of re-bleeding after successful endoscopic therapy for peptic ulcers.

## Materials and methods

We conducted a prospective, comparative study at a tertiary care hospital in Pakistan from January 1, 2018 to June 30, 2019. We obtained approval from the Ethical Review Committee of the institution. Informed consent was received from all participants.

All patients presenting to the gastroenterology unit with an active complaint of UGIB secondary to PUD during the study period were included. Patients younger than 18 years of age, those who were unwilling to participate in the study, those who had unsuccessful endoscopy or very low risk of re-bleed (flat-pigmented with clean base ulcers), those with coagulopathy, liver cirrhosis, Mallory-Weiss tear, or uremia, and those with suspicion of malignant ulcers were excluded from the study.

After stabilizing the patients hemodynamically, gastroesophageal endoscopic ultrasound was performed within 24 hours of presentation. Before the procedure, all patients were given IV pantoprazole (80 mg IV stat followed by 8-mg per hour infusion). After the endoscopic ultrasound, patients were randomly divided into two groups by coding their patient registration numbers; odd codes were grouped together as group A and even codes as group B. Group A received 80 mg IV pantoprazole as an infusion over 30 minutes after endoscopy followed by 8-mg IV per-hour infusion for the next three days. Group B received 80 mg oral pantoprazole after endoscopy followed by 80 mg twice daily for the next three days.

After 72 hours of endoscopic ultrasound, all patients of both the groups were shifted to oral pantoprazole 40 mg twice daily. Hemoglobin (Hb) levels were checked every 12 hours. Packed cells were transfused in case Hb was lower than 7 mg/dL in young patients (<50 years) or lower than 9 mg/dL in older patients (>50 years). Re-bleeding was assessed on the basis of hematemesis, orthostatic hypotension [supine and sitting blood pressure (BP)], or hemodynamic instability (respiratory rate and pulse). If re-bleeding was suspected, urgent re-endoscopy was done and a similar protocol of oral or IV pantoprazole was repeated. On discharge from the hospital, all patients were prescribed oral pantoprazole 40 mg twice daily. All patients were advised for follow-ups at the end of the month or earlier in case of any complaints.

Data collection was performed in the form of a questionnaire which comprised patient demographics, previous UGIB history, history of NSAIDs and/or aspirin intake, melena, hematemesis, quality and quantity of blood products transfused, duration of hospital stay, endoscopic outcomes, need for re-endoscopy or surgery, and rate of mortality until the end of the one-month follow-up after endoscopy. All the data thus collected were subjected to statistical analysis using Statistical Package for the Social Sciences (SPSS) software version 23.0 (IBM, Armonk, NY). Mean and standard deviation (SD) were calculated for quantitative variables. Frequency and percentage were calculated for categorical variables. A chi-square test was applied to test the significant difference between the two groups. A p-value of ≤0.05 was considered statistically significant.

## Results

We included 200 patients in the study. Group A had 96 (48%) patients, and group B included 104 (52%). There were 59 (61.5%) males and 37 (38.5%) females. The mean age of the study sample was 56.3 ±4.1 years. The demographic and clinical characteristics of both groups are compared below in Table 1.

**Table 1:** Demographic characteristics and clinical history of patients in IV and oral pantoprazole groups IV: intravenous; NSAIDs: non-steroidal anti-inflammatory drugs; SD: standard deviation

Baseline characteristics	Group A (IV pantoprazole) (n = 96)	Group B (oral pantoprazole) (n = 104)
Age in years, mean ±SD	57.1 ±3.3	58.1 ±3.9
Gender, n (%)		
Male	59 (61.5)	62 (56.9)
Female	37 (38.5)	42 (40.4)
Smoking, n (%)	33 (34.4)	36 (34.6)
Drug history, n (%)		
Aspirin or NSAIDs	69 (71.9)	75 (72.1)
Clopidogrel	12 (12.5)	12 (11.5)
Warfarin	13 (13.5)	10 (9.6)
Baseline hemoglobin, mg/dL, mean ±SD	8.1 ±1.3	8.2 ± 1.9
Melena, n (%)	75 (78.1)	93 (89.4)
Hematemesis, n (%)	52 (54.2)	56 (53.8)

Endoscopy was done in all patients. Bleeding gastric ulcers were more commonly seen in group A (42% vs. 38%), and 61.5% of the patients in each group had bleeding duodenal ulcers. Non-bleeding visible vessel was significantly more common in group A (52% vs. 34%), and spurting was significantly more common in group B (11% vs. 8%) (Table 2).

**Table 2:** Endoscopic findings in patients of IV and oral pantoprazole groups IV: Intravenous

Endoscopy findings	Group A (IV pantoprazole) (n = 96)	Group B (oral pantoprazole) (n = 104)	P-value
Gastric ulcer, n (%)	40 (41.7)	39 (37.5)	0.54
Duodenal ulcer, n (%)	59 (61.5)	64 (61.5)	0.281
Adherent clot, n (%)	30 (31.3)	29 (27.9)	0.99
Oozing, n (%)	27 (28.1)	29 (27.9)	0.96
Non-bleeding visible vessel, n (%)	50 (52.1)	36 (34.6)	0.01
Spurting, n (%)	8 (8.3)	11 (10.6)	<0.001

Clinical and biochemical characteristics of the patients after endoscopy were compared. From 24 hours of receiving medication onwards, the IV pantoprazole group showed a significant improvement in Hb levels (p: 0.01); the group also showed improvement in supine systolic BP at 48 hours (p: 0.04) and in diastolic at both 12 and 48 hours as compared to the oral pantoprazole group (p: 0.05). BP at sitting position was significantly better in group A (p: ≤0.05). Group B had higher respiratory and pulse rates (p: ≤0.05) (Table 3).

**Table 3:** Post-endoscopy biochemical and clinical characteristics of patients in IV and oral pantoprazole groups BP: blood pressure; IV: intravenous; SD: standard deviation

Patient characteristics	Group A (IV pantoprazole) (n = 96)	Group B (oral pantoprazole) (n = 104)	P-value
Hemoglobin, mg/dL, mean ±SD			
12 hours after endoscopy	7.4 ±2.3	7.1 ±3.1	0.44
24 hours after endoscopy	7.9 ±1.5	7.3 ±1.9	0.01
48 hours after endoscopy	8.7 ±1.1	8.0 ±3.0	0.03
72 hours after endoscopy	9.1 ±2.5	8.7 ±1.7	0.003
Supine BP, mmHg, mean ±SD			
Systolic at 24 hours after endoscopy	100.4 ±15.7	100.1 ±18.3	0.90
Systolic at 48 hours after endoscopy	117.4 ±11.7	113.9 ±13.2	0.04
Diastolic at 12 hours after endoscopy	72.7 ±5.6	68.4 ±8.7	<0.001
Diastolic at 48 hours after endoscopy	70.1 ±5.1	72.4 ±10.8	0.05
Sitting BP, mmHg, mean ±SD			
Systolic at 24 hours after endoscopy	102.7 ±7.3	98.5 ±6.1	<0.001
Systolic at 48 hours after endoscopy	110.7 ±0.8	109.7 ±0.8	<0.001
Diastolic at 12 hours after endoscopy	68.3 ±10.4	65.7 ±7.3	0.04
Diastolic at 48 hours after endoscopy	72.7 ±2.4	70.1 ±4.3	<0.001
Respiratory rate per minute, mean ±SD			
At 12 hours after endoscopy	23.1 ±2.4	26.4 ±1.8	<0.001
At 48 hours after endoscopy	19.7 ±1.8	22.7 ±2.3	<0.001
Pulse per minute, mean ±SD			
At 12 hours after endoscopy	97.4 ±15.7	99.1 ±17.1	0.46
At 48 hours after endoscopy	80.3 ±8.6	89.4 ±9.5	<0.001

The mean volume packed cells transfused in group A was 114.2 ±20.1 ml as compared to 174.5 ±31.4 in group B (p: <0.001). Mean duration of hospital stay was comparable between the two groups and the differences were not significant (3.5 ±1.3 days in group A vs. 3.7 ±1.3 days in group B; p: 0.27). Outcomes were assessed in terms of need for repeat endoscopy, re-bleeding events, and mortality rates. There were no differences between the outcomes of the two study groups (Table 4).

**Table 4:** Study outcomes in patients in IV and oral pantoprazole groups IV: intravenous

Outcome	Group A (IV pantoprazole) (n = 96)	Group B (oral pantoprazole) (n = 104)	P-value
Mortality, n (%)	8 (8.3)	6 (5.8)	0.58
Re-bleeding, n (%)	4 (4.2)	7 (6.7)	0.42
Repeat endoscopy, n (%)	5 (5.2)	4 (3.8)	0.64

## Discussion

The results of the study showed no difference between the two groups in terms of reduction in the incidence of re-bleeding. Patients in both oral and IV pantoprazole groups had similar rates of re-bleeding, duration of hospital stay, amount of transfused blood, and instances of re-endoscopy; the rate of mortality until the end of the one-month follow-ups after endoscopy was also similar for both groups. Similar findings have been found in previous literature [10].

In a study by Tsai et al., oral and IV route of pantoprazole was compared in high-risk PUD patients after therapeutic endoscopy, and they also showed similar effects for both routes [11]. Other studies have also demonstrated that there was no statistically significant difference between two routes of administration of PPIs in terms of re-surgery, re-bleeding, mortality rates, hospital stay, and need for blood transfusion [9,12,13]. Almost all the studies that compared the two routes of PPI administration showed that they were almost equally effective and revealed no statistically significant difference between the two [14,15]. A recent study conducted with 44 patients in the IV PPI group and 41 in the oral PPI group after successful endoscopy for prevention of re-bleeding found that the rate of re-bleeding, duration of hospital stay, and need for transfusion were comparable in both groups [16].

Some recent guidelines recommend treating high-risk patients after endoscopy with IV bolus of PPIs followed by continuous infusion [17,18]. Other guidelines have not specified any route of PPI administration in their recommendations [19]. In a randomized controlled trial, oral PPIs showed similar 24-hour intragastric pH as compared to IV bolus infusion. However, the IV PPI group reached a mean pH of 6 one hour earlier than the oral PPI group [16]. In light of the similarity in 24-h pH monitoring between both routes of administration, oral PPIs are expected to largely take over IV therapy [16]. Two studies conducted in Asia demonstrated that oral PPI therapy adjunct to endoscopy reduced re-bleeding risk by 14-50% [20,21].

When compared to oral therapy, the IV route of PPI administration is more expensive, difficult to manage, and needs professional supervision in terms of nursing care and clinical monitoring [22,23]. Pakistan being a resource-limited country, the cost of therapy is a huge factor for both healthcare providers and the patients while choosing a medical treatment. Oral PPIs allow for cost-cutting without compromising treatment efficacy and outcomes. Spiegel et al. compared three routes of PPI administration in terms of clinical and economic outcomes. They demonstrated that oral PPIs were more cost-effective when compared to IV [24].

## Conclusions

We are able to conclude that there is no statistically significant difference between oral and IV routes of pantoprazole administration in the prevention of rebleeding when used after successful therapeutic endoscopy in patients with bleeding PUD. However, we recommend that oral PPIs be favored over the IV variant in patients as they are easier to administer and more cost-effective.
